RETRACTED

# Contrast and Synthetic Multiexposure Fusion for Image Enhancement

**DOI:** 10.1155/2021/2030142

**Published:** 2021-09-03

**Authors:** Marwan Ali Albahar

**Affiliations:** Umm Al Qura University, College of Computer Science in Al-Leith, Mecca, Saudi Arabia

## Abstract

Many hardware and software advancements have been made to improve image quality in smartphones, but unsuitable lighting conditions are still a significant impediment to image quality. To counter this problem, we present an image enhancement pipeline comprising synthetic multi-image exposure fusion and contrast enhancement robust to different lighting conditions. In this paper, we propose a novel technique of generating synthetic multi-exposure images by applying gamma correction to an input image using different values according to its luminosity for generating multiple intermediate images, which are then transformed into a final synthetic image by applying contrast enhancement. We observed that our proposed contrast enhancement technique focuses on specific regions of an image resulting in varying exposure, colors, and details for generating synthetic images. Visual and statistical analysis shows that our method performs better in various lighting scenarios and achieves better statistical naturalness and discrete entropy scores than state-of-the-art methods.

## 1. Introduction

Currently, several hardware- and software-based solutions are enhancing the quality of images captured with smartphone cameras. Image quality enhancement is still a big challenge under high dynamic range and poor lighting conditions. Various software techniques have been proposed to improve the visual quality of images in these conditions. The goal is to enhance the visibility of low-lighting parts of the image while keeping others' quality intact. Histogram equalization techniques [1–4] try to improve the contrast and visibility of photos. Likewise, adaptive gamma correction techniques [5, 6] have also been proposed to improve contrast in images. However, these techniques can over-enhance images in bright regions and under-enhance them in dark regions. Neural network- (NN-) based techniques [7, 8] have also been developed, which perform specific image enhancement tasks. However, these techniques have some intrinsic limitations, including slow processing speed and huge memory requirements. Additionally, training NNs requires a large amount of training data, which is not easily available or does not generalize well to different scenarios, rendering their unsuitability for a variety of smartphone-related tasks. Exposure fusion [9, 10] is yet another technique that improves the quality of an image by combining multiple low dynamic range images of varying exposures and fuses the best parts of each image. However, this technique introduces artifacts in the presence of motion blur in the image stack. It is nearly impossible to capture a static burst of images using smartphone cameras. Burst image alignment techniques have been proposed to mitigate this problem. Furthermore, to maximize the benefits of exposure fusion, various methods for generating pseudo-multi-exposure images from a single image have been proposed in [11–13]. As a result, there is no single method for creating high-quality, artifact-free images.

- We propose a novel method of generating synthetic multiexposure images by applying gamma corrections to input images with different gamma parameters and processing these images with existing image enhancement techniques.
- The segmentation of the input image is divided into various regions based on its luminosity. This results in more exposure in generated images as each generated image focuses on a specific region during the enhancement process.
- We extend this method to create a four-step image enhancement pipeline, which utilizes contrast enhancement and exposure fusion to generate an output image.

RETRACTED

The proposed solution is applied to synthetic natural images to test its performance. The corresponding comparative experiment results confirm that our methodology is more robust to different imaging scenarios and produces better visual quality than the existing methods.

The rest of this article is organized as follows: Section 2 discusses related work; Section 3 elaborates the proposed structure in detail; Section 4 analyzes the experimental results; and Section 5 concludes this article.

## 2. Related Work

There are several techniques for image enhancement that improve the visual quality of images. Some most common techniques work on low light and high dynamic range scenarios. In darker regions, visual quality can be improved by increasing luminosity while keeping the noise minimal and avoiding overblowing details in the brighter regions. There exist various approaches to solve this problem ranging from neural network-based approaches [7, 8], to gamma correction [5, 6], burst image alignment [14–16], and retinex-based methods [17, 18]. In [19], a single-image dehazing solution based on the adaptive structure decomposition-integrated multi-exposure image fusion (PADMEF) was proposed to effectively eliminate the visual degradation caused by haze without the physical model inversion of haze formation. The authors of [20] proposed using a novel image dehazing framework that is based on the fusion of artificial multiexposure images. The proposed algorithm can produce high-visibility images by effectively and efficiently mitigating the effects of adverse haze on the environment. The proposed algorithm could be used to create images without requiring any modifications to existing imaging devices.

RETRACTED

Most of them are some form of contrast enhancement techniques. In the current work, our aim is to develop a novel method that is compatible with smartphones. Therefore, it has to be resource-efficient in terms of computational and memory requirements. Our proposed technique is thus based on histogram and synthetic exposure fusion-based techniques.

### 2.1. Histogram-Based Methods

Most common contrast enhancement technique is histogram equalization [1]. The goal of this technique is to make the histogram of the image uniformly distributed to increase contrast. Various extensions of this method have been proposed that usually perform global or local histogram equalization. Contrast limited adaptive histogram equalization (CLAHE) [2] is a commonly used local contrast enhancement technique, which divides the image into several tiles. Contrast transformation for each tile is performed. Afterward, these tiles are combined using bilinear interpolation to avoid unnatural boundaries between tiles. Joint histogram equalization approaches have also been proposed, which combine both global and local approaches. Joint histogram equalization (JHE) [4] uses an average image along with the original image to create a two-dimensional joint histogram. A two-dimensional cumulative distribution function is then computed, which generates the contrast-enhanced output pixel value. Global and local contrast adaptive enhancement for nonuniform illumination color images (GLFs) [3] also utilize both local and global contrast enhancement. The input image is linearly stretched, globally and locally enhanced, further merged, and hue preservation is performed. Global contrast enhancement is performed by obtaining a modified histogram, which is closest to a uniform histogram. For local contrast enhancement, CLAHE [2] is used. Hue preservation equations from Nikolova and Steidl [21] are used as shown in equations (1) and (2). These enhanced images are merged by using weighted sums. Weight maps are generated by applying the Laplacian filter and fitting pixel intensity to the Gaussian curve:

(1) $$\begin{array}{c} I_{h}≔\left\{\begin{array}{cc} \theta , & \text{if }c_{b}\leq c_{g},\\ 360^{o}-\theta , & \text{if }c_{b}>c_{g}, \end{array}\right. \end{array}$$

where *c*_*b*_, *c*_*g*_, and *c*_*r*_ are the blue, green, and red channels of the image for which the process is performed, and

(2) $$\begin{array}{c} \theta =\frac{\left(1/2\right)\left(\left(c_{r}-c_{g}\right)+\left(c_{r}-c_{b}\right)\right)}{{\left({\left(c_{r}-c_{g}\right)}^{2}+\left(c_{r}-c_{b}\right)\left(c_{g}-c_{b}\right)\right)}^{2}}. \end{array}$$

RETRACTED

### 2.2. Synthetic Exposure Fusion

Exposure fusion [9] is a technique used to combine multiple low dynamic range images of the same scene to get a single high quality image. The best parts from the input sequence are taken and fused together seamlessly. However, there are strict requirements for this technique to work correctly. Input image sequences must have varying exposures, and the scene must be static, not usually possible with cameras when taking multiple images of the same scene. To counter this problem, various techniques have been proposed recently, which generate multiple synthetic images with varying exposures and then fuse them together using exposure fusion. Bio-inspired Multiexposure fusion framework (BioMEF) [13] proposes a four-step procedure for this task. In the first step, the required number of synthetic images is determined. In the second step, the camera response model is used to generate synthetic images. In the third step, weight maps are assigned to these images, combined in the fourth step of the procedure. Scene segmentation-based luminance adjustment (SSLA) [12] also provides an approach to generate multiple synthetic exposure images from a single image. Gamma correction with a fixed value of 2.2 is applied to the input image. In the subsequent step, local contrast enhancement is applied to the input image. Then, the luminosity values of this image are sorted and divided into *M* equal regions. The enhancement factor is calculated from each region, which is then used to scale the existing image to generate synthetic images. Inverse gamma correction is performed, and then these images are fused using exposure fusion.

### 2.3. Machine Learning-Based Image Enhancement Techniques

Numerous works exist based on machine learning, which can be further categorised in unsupervised and supervised image enhancement techniques [22]. The unsupervised works model the data using various classifiers such as K-mean [23], hierarchical clustering [24], and EM algorithm [25]. The prominent works based on unsupervised techniques consist histogram equalization [2, 26–29], retinex-based enhancement [30–34], visual cortex neural network-based enhancement [35–38], and Rybak model [39, 40]. In unsupervised-based image enhancement techniques, most of the methods are based on convolutional neural network (CNN) consisting generative adversarial [41, 42] and power-constrained contrast enhancement (PCCE) [43] techniques. The most commonly used techniques are based on reinforcement learning [44, 45], U-Net [46], fully convolutional networks (FCN) [7, 47], multilevel features fusion methods [48–53], and retinex-based deep learning methods. The unsupervised techniques mainly focus on one dimension of the image enhancement. Some works focus on exposure correction of dark images and denoising, while other focus on white balancing and dehazing. Similarly, the supervised-based methods are related to one of the modules. Those supervised learning-based methods that incorporated multiple image enhancement dimensions are computationally expensive and required a large amount of data. Our focus is on contrast enhancement of over and underexposed images along with dark and bright images in this work. The proposed techniques are time efficient and have outperformed the existing methods for enhancing various exposure images. In this paper, we propose a novel way of generating multiple synthetic exposure fusion by applying gamma corrections to the input image based on its luminosity values before using image enhancement techniques. In this way, we force the image enhancement techniques to primarily target a specific under or overexposed region of the image, which results in higher variation in synthetically generated images. We propose an image enhancement pipeline that is more robust to different lighting scenarios and works well to improve image quality.

RETRACTED

## 3. Proposed Methodology

The proposed image enhancement pipeline consists of four parts: image analysis, gamma parameter calculation, synthetic image generation, and exposure fusion. An overview of the proposed method is given in Figure 1 and further, the complete pipeline is explained step by step.

### 3.1. Overview

To increase the robustness of our method to different imaging scenarios, input images are divided into three categories: normal, dark, and extreme. Dark images are those, which are taken in very low lighting conditions. Intense images have regions that are underexposed and other regions, which are overexposed or have correct exposure. These two types of images are usually over or under enhanced by existing methods hence the need for categorization. All other images are part of the normal category. This categorization is done in the first step, i.e., image analysis. In the next step, parameters for gamma correction are determined. The image is divided into three regions based on its luminosity. These regions determine the four gamma parameters used in the subsequent step. In the next step, multiple synthetic images are generated. The input image is subjected to gamma corrections using generated gamma parameters. The first three of these images are subject to contrast enhancement based on GLF [3]. This results in aggressive enhancement. The fourth image is subject to a modified version of SSLA [12]. This algorithm improves image quality along with retaining much information from the original image. This is especially necessary for dark and extreme images. In the final step, synthetic images are merged together using exposure fusion.

RETRACTED

### 3.2. Image Analysis

Images with very low light conditions or large exposure differences among regions are susceptible to over or under enhancements. To avoid this, input images are divided into three categories: normal, dark, and extreme. luminance channel *L* of *n* images is extracted. If the mean value of intensities of *L* is less than 85, the image is classified as dark where this number is equal to one-third of the sum of the maximum value in each channel. Next, we check whether the image lies in the extreme category. For this, the intensities are divided into two regions: bright and dark. If the intensity at a pixel is greater than 127, it is considered bright. Otherwise, it is considered dark. This number is computed as half of the maximum value in a channel. Similarly, if the mean of dark pixels is less than 28 and the ratio between dark and bright pixels is between 20 and 80, the image lies in the category of extreme images. If an image lies in both dark and extreme categories, it is treated as an extreme image. All other images are classified as normal. To speed up this process, we reduce the size of the image by 95 percent as the overall composition of the image remains the same even when downsampled, and resizing do not affect the result. The value 95 is considered the standpoint and is determined empirically. As we go down this point, degradation and information loss occur in the respective images.

### 3.3. Gamma Parameter Calculation

In this step, we again work with the luminance channel *L* that is divided into three equal regions based on pixel intensity values. Let *L*_*s*_ be an array of sorted luminosity values of size *n*. We get the length *k* of each region by

(3) $$\begin{array}{c} \left[H\right]k=\frac{\max\left(L_{s}\right)-\min\left(L_{s}\right)}{3}. \end{array}$$

First *k* entries of *L*_*s*_ are assigned to the first region, the next *k* entries to the second region, and the third region. Afterward, gamma parameters for all three regions are calculated using the following equations:

(4) $$\begin{array}{c} v_{i}=\frac{1}{\left|E\right|}\sum_{p\in R_{i}}\log\left(\max\left(p,ɛ\right)\right), \end{array}$$

(5) $$\begin{array}{c} \alpha_{i}=\frac{v_{i}}{2.2}, \end{array}$$

where *R*_*i*_ is the *i*-th region, *ϵ* is assigned to a small value to avoid singularities where *p*=0 and *α*_*i*_ is the calculated *i* -th parameter. This gives us the first three parameters. In the next step, the generated parameters are further adjusted to give the best visual and statistical results, and the value of the fourth parameter is also assigned. These adjustments are defined in Table 1. This process gives us the parameters to be used in the next phase for synthetic image generation. Moreover, it is worth mentioning that these parameters sometimes give degraded results; therefore, the parameters are sometimes used with a slight standard deviation of ±0.5, which are mentioned in detail during the process. Similarly, image reduction is also performed here, as in the previous step, to improve the performance of our process.

RETRACTED

### 3.4. Synthetic Image Generation

In this step, multiple synthetic images are generated from the single-source image. The previously calculated parameters are used to perform gamma corrections on the input image to generate four different images. Each gamma-corrected image corresponds to a different level of exposure. Two images are overexposed, whereas the other two are underexposed to varying degrees. The first three gamma-corrected images are passed to the modified GLF module. This module consists of two parts: local contrast enhancement and global contrast enhancement. We utilize JHE [4] for global contrast enhancement while other implementation details remain the same as the original work. This module aggressively enhances the contrast of the image. However, this could result in unwanted artifacts and too much deviation from original colors, especially in dark and extreme images. To maintain closeness to the original image, we also use a modified version of SSLA. We use the second approach defined in [12] to segment the image into seven parts. We also resize the image to a very small size while calculating the luminance scaling factor to speed up the process. Moreover, the original implementation [4] performs gamma correction of 2.2, which is not suitable in all scenarios. Instead, we pass the already gamma-corrected image with gamma parameter *α*_4_. Similar to the original implementation, we perform inverse gamma correction with value *α*_4_ before fusing the generated images. We avoid the local contrast enhancement step as it does not increase the performance measures and increases the overhead of the contrast enhancement step. This module results in an enhanced image, which is much closer to the original image and avoids enhancements. At the end of this step, we have obtained four synthetically generated multiexposure images.

### 3.5. Exposure Fusion

In the last part of our image enhancement pipeline, we use exposure fusion to combine the synthetic images to generate the final output image. Exposure fusion is a process that takes multiple input images of the same scene, with slight variation in contrast or brightness, selects the best pixels from all the images, and generates a single image of the same scene out of the input images. Technically, it assigns weights to each pixel based on the local properties and combines them in a single-output image. Next, all the four synthetic images and the input image are merged together using exposure fusion to generate a high-quality image.

RETRACTED

## 4. Results and Comparison

We tested our method on images with different lighting scenarios. We used VV dataset [54] to test our method. This dataset contains 24 images under extreme lighting conditions. Each image in this dataset has a part, which is correctly exposed, while other parts are extremely under or overexposed. Moreover, we generated our own dataset consisting of 44 images having a variety of different lighting conditions, including low light images, high dynamic range scenes, properly exposed scenes, and extreme lighting conditions similar to the VV dataset [54]. We compared our methodology to CLAHE [2], AGCWD [5], SSLA [12], GLF [3], and BioMEF [13].

### 4.1. Subjective Analysis

In this subsection, we provide a visual comparison of our methodology to other methodologies and compare results. We perform this visual analysis under different lighting conditions.  Figure 2 shows that our methodology works quite well under extremely low lighting conditions. Colors and details are better than other methodologies. Only GLF [3] comes close to match the visual quality of our method. However, our techniques illustrate that the input image has more salient features which is visible to the naked eye, as can be seen from Figure 2(g). Specifically, if we compare the corners of the GLF with the proposed method's output, it can be clearly seen that the result of the proposed method is more evident and clearly visible.

Figure 3 depicts a high dynamic range scene where our methodology retains a good balance between underexposed regions and retaining color and details in the remaining regions of the original image. In this comparison, the output of the GLF technique is almost similar to the proposed techniques with subtle variations and differences. Upon close analysis, the proposed technique has better output than the rest of the techniques, as can be seen from Figure 3.

The extreme scene in Figure 4 shows that our method has more vivid colors in the foreground and the sky. Again GLF seems to come close, but it does produce some unwanted artifacts, such as a pink box of a pixel in the middle of the image.

RETRACTED

Under normal lighting scenario depicted by Figure 5, our method improves visual quality the most while retaining details. Colors have started to fade in GLF, which has been performing quite well so far. SSLA and BioMEF perform well, but there is a bit hazing effect. The performance of AGCWD is comparatively good; however, it overexposes some parts of the image.

In the overexposed scenario shown in Figure 6, AGCWD represents good colors but does not deal with overexposed parts of the image. Here, the GLF shortcomings are also revealed as it is not well suited for highly or adequately exposed scenes. The hazing effect in BioMEF is also highlighted in this scenario. Hence, our methodology again shows a good balance between colors and details.

Visual comparison in different scenarios proves the robustness of our method as compared to existing state-of-the-art techniques. Also, the visual quality steadily remains the best in all scenarios.

### 4.2. Statistical Analysis

For statistical analysis, discrete entropy (DE) [55] and statistical naturalness measure (SNM) [56] are used to compare the proposed method with the existing state-of-the-art techniques. Discrete entropy shows the richness of details in the image. However, this measure can be affected by over enhanced images, which score higher in this category. Therefore, we also introduce statistical naturalness measures to keep check of over enhancements. Sum of discrete entropy and statistical naturalness measure scores of all images in respective datasets are shown in Tables 2 and 3. A higher score means a better result.

The highest values are shown in bold, while the second highest is shown in italics.

Our method achieves the highest discrete entropy and statistical naturalness measure scores on both datasets. This confirms our observations during the visual comparison. The proposed method improves quality and retains many details better than the existing techniques in all tested scenarios while avoiding over or under enhancements.  Table 4 shows the time taken by each method to generate results for our dataset. SSLA and GLF have code available in Matlab, whereas AGCWD, BioMEF, and CLAHE have implementations available in python; however, our method runs on C++. Although programming languages affect this time comparison, the comparison demonstrates a general idea about the speed of algorithms. We see that all methods other than BioMEF generate results in a respectable amount of time.

Worth noting that in the proposed method, we do not perform any kind of noise reduction that is why in low-lighting conditions, it may produce noisy images. In most cases, the utilized contrast enhancement techniques work well but may produce some unwanted artifacts, as shown in Figure 7.

RETRACTED

## 5. Conclusion

In this work, we have proposed a novel procedure for generating synthetic multi-exposure fusion images with much more variation in exposure than the existing methods. This is achieved by first optimizing the gamma correction parameters concerning the luminosity of the input image. Then, gamma correction with optimized parameters is applied on each image that is further enhanced using existing contrast enhancement techniques. The use of differently gamma-corrected images before enhancement ensures that each generated synthetic image focuses on a specific exposure region. This results in a higher variation of exposure, color, and details in generated images. We extended this work to create an image enhancement pipeline that is robust to different lighting scenarios. The visual and statistical comparison shows that our methodology improves the quality of the image while retaining details in all multiple imaging scenarios. In the current work, we have utilized two different methods for enhancement. In the future, we intend to use a single more robust contrast enhancement technique. Similarly, the number of generated gamma parameters and their defined adjustments will be looked upon in the future for better results.

## Figures and Tables

**Figure 1:** Steps involved in the proposed pipeline technique, where an input image is categorised into one of three categories (normal, dark, and light). Furthermore, the gamma parameters are calculated, and in the next step, four synthetic images are generated based on these gamma parameter values. In the last step, all the synthetic images and the input image are merged using synthetic multi-exposure fusion, which results in a high-quality image.

**Figure 2:** Under low-light scenario input image and processing with state-of-the-art methods along with comparison with the proposed technique. (a) Original. (b) CLAHE. (c) AGCWD. (d) SSLA. (e) GLF. (f) BioMEF. (g) Proposed.

**Figure 3:** High dynamic range scene. (a) Original. (b) CLAHE. (c) AGCWD. (d) SSLA. (e) GLF. (f) BioMEF. (g) Proposed.

**Figure 4:** Extreme lighting scene. (a) Original. (b) CLAHE. (c) AGCWD. (d) SSLA. (e) GLF. (f) BioMEF. (g) Proposed.

**Figure 5:** Normal scenario. (a) Original. (b) CLAHE. (c) AGCWD. (d) SSLA. (e) GLF. (f) BioMEF. (g) Proposed.

**Figure 6:** Overexposed scene. (a) Original. (b) CLAHE. (c) AGCWD. (d) SSLA. (e) GLF. (f) BioMEF. (g) Proposed.

**Figure 7:** Failure case. (a) Original. (b) Proposed.

**Table 1:** Gamma parameters adjustment.

Parameter	Normal	Dark	Extreme
*α*_0_	*α*_0_	1	*α*_1_
*α*_1_	(1/*α*_1_)	*α*_1_	*α*_2_
*α*_2_	(1/*α*_2_)	(1/*α*_2_)	(1/*α*_2_)
*α*_4_	*α*_0_	(1/*α*_1_)	*α*_2_

RETRACTED

**Table 2:** Comparison of discrete entropy (DE) and statistical naturalness measure (SNM) on our dataset.

	DE	SNM
CLAHE	289.86	14.15
AGCWD	282.16	13.23
SSLA	209.82	24.84
GLF	325.18	25.64
BioMEF	289.74	20.64
Proposed	**332.76**	**26.93**

The highest values are shown in bold, while the second highest is shown in italics.

**Table 3:** Comparison of discrete entropy (DE) and statistical naturalness measure (SNM) on the VV dataset.

	DE	SNM
CLAHE	164.78	7.31
AGCWD	163.19	10.28
SSLA	171.77	14.85
GLF	176.25	13.92
BioMEF	169.22	12.93
Proposed	**178.91**	**16.75**

**Table 4:** Time comparison of various methods in seconds.

Techniques	Time (s)
CLAHE	1.01
AGCWD	9.29
SSLA	32.38
GLF	50.10
BioMEF	276.59
Proposed	32.21

## Data Availability

Datasets used to support the findings of this study are included within the article.
